RETRACTED

# Automatic Detection of High-Frequency Oscillations Based on an End-to-End Bi-Branch Neural Network and Clinical Cross-Validation

**DOI:** 10.1155/2021/7532241

**Published:** 2021-12-28

**Authors:** Zimo Liu, Penghu Wei, Yiping Wang, Yanfeng Yang, Yang Dai, Gongpeng Cao, Guixia Kang, Yongzhi Shan, Da Liu, Yongzhao Xie

**Affiliations:** ^1^Key Laboratory of Universal Wireless Communications, Ministry of Education, Beijing University of Posts and Telecommunications, No. 10 Xitucheng Road, Haidian District, Beijing 100876, China; ^2^Department of Neurosurgery, Xuan Wu Hospital, Capital Medical University, No. 45 Changchun Street, Xicheng District, Beijing 100053, China; ^3^Beijing Baihui Weikang Technology Co., Ltd., Beijing 100083, China

## Abstract

Accurate identification of high-frequency oscillation (HFO) is an important prerequisite for precise localization of epileptic foci and good prognosis of drug-refractory epilepsy. Exploring a high-performance automatic detection method for HFOs can effectively help clinicians reduce the error rate and reduce manpower. Due to the limited analysis perspective and simple model design, it is difficult to meet the requirements of clinical application by the existing methods. Therefore, an end-to-end bi-branch fusion model is proposed to automatically detect HFOs. With the filtered band-pass signal (signal branch) and time-frequency image (TFpic branch) as the input of the model, two backbone networks for deep feature extraction are established, respectively. Specifically, a hybrid model based on ResNet1d and long short-term memory (LSTM) is designed for signal branch, which can focus on both the features in time and space dimension, while a ResNet2d with a Convolutional Block Attention Module (CBAM) is constructed for TFpic branch, by which more attention is paid to useful information of TF images. Then the outputs of two branches are fused to realize end-to-end automatic identification of HFOs. Our method is verified on 5 patients with intractable epilepsy. In intravalidation, the proposed method obtained high sensitivity of 94.62%, specificity of 92.7%, and F1-score of 93.33%, and in cross-validation, our method achieved high sensitivity of 92.00%, specificity of 88.26%, and F1-score of 89.11% on average. The results show that the proposed method outperforms the existing detection paradigms of either single signal or single time-frequency diagram strategy. In addition, the average kappa coefficient of visual analysis and automatic detection results is 0.795. The method shows strong generalization ability and high degree of consistency with the gold standard meanwhile. Therefore, it has great potential to be a clinical assistant tool.

RETRACTED

## 1. Introduction

Accurate localization of epileptogenic zone (EZ) is the key to the success of preoperative assessment of patients with drug-refractory epilepsy [1–3]. Detection of high-frequency oscillation (HFO) signal with a frequency of 80–500 Hz is of great significance for accurate localization of EZ, since as a biomarker of EZ [4–7], a good prognosis is highly correlated with surgical resection of the channel with a high incidence of HFOs [4, 8]. HFOs are spontaneous electroencephalogram patterns, which reflect the synchronous transient of neurons [9]. They are divided into three types according to frequency: Rs (Ripples, 80–250 Hz), FRs (Fast Ripples, 250–500 Hz), and VHFOs (very high-frequency oscillations, 1000–2500 Hz) [10, 11]. At present, clinicians' visual analysis of HFOs based on long-term stereoelectroencephalography (SEEG) and video recordings is considered as the gold standard for clinical diagnosis [12–15]. However, one patient usually needs to be continuously monitored for several days to a week, so manual analysis of such a huge amount of data is beyond the reach of clinical manpower. In addition, visual analysis is affected by doctors' subjective factors, leading to unavoidable miss and wrong labels [16]. Therefore, it is of great practical significance to explore the automatic detection method of HFOs, which can provide more objective basis for clinicians with reduction of manpower.

Many HFOs automatic detectors have been reported in different studies. The conventional method of HFOs detection is usually based on either the band-pass signal or the time-frequency diagram. In terms of signal, single-step detection methods with different characteristics of Teager energy operator, wavelet entropy, fuzzy entropy, short-time energy, and so on have been studied in the past 10 years [17–24]. However, it is difficult for these methods to distinguish HFOs from some artifacts, such as spikes, pulse-like artifacts, and signals with harmonics [20]. To alleviate this problem, two-stage methods are proposed to further explore the signal characteristics by adding a supervised classifier or an unsupervised clustering after an initial detector [25–29]. Specifically, real HFOs can be identified from the candidate events isolated from background activities by a stacked CNN [28] or a stacked denoising autoencoder [29], while in terms of time-frequency diagram, the two-stage automatic detection paradigm has always been used. In particular, it is the simple 2d-CNN structure that is often used as a time-frequency image feature extractor after an initial detector [25, 30–32]. However, it is still a challenge to fully learn useful information worth attention in either signals or time-frequency images.

RETRACTED

Although the above studies have been implemented and their effectiveness is verified to some extent, there are still some challenges to overcome. In clinical diagnosis, multimodal data is often used by clinicians to achieve an accurate preoperative assessment [33–35]. In EEG analysis, two different modalities of signal waveform and time-frequency analysis image contain abundant information, respectively, which needs neurologists' comprehensive analysis [36]. But, few studies have taken both of the data forms into account. Besides, previous studies seldom paid attention to both the temporal dimension characteristics and the spatial morphology characteristics of signals, and few researchers conducted deep analysis about which information in time-frequency images is worthy attention and which is not. So, the single analysis perspective and simple model design of previous methods resulted in the following 3 challenges: (1) insufficient modal of input data, (2) insufficient learning of temporal and spatial morphological features of EEG signal, and (3) insufficient learning of the features in time-frequency diagram.

To address aforementioned challenges, this paper proposes an HFOs automatic detection method based on an end-to-end bi-branch fusion model, which not only can integrate the advantages of both modals' data but also can explore more abundant signal or image information from multiperspectives. With the filtered band-pass signal (signal branch) and time-frequency image (TFpic branch) as the input of the model, two backbone networks for deep feature extraction are established, respectively. Specifically, a hybrid model based on ResNet1d and LSTM is designed for signal branch, while a ResNet2d with a CBAM block is constructed for TFpic branch. Then the outputs of two branches are fused to realize end-to-end automatic identification of HFOs. Our proposed method is evaluated by using clinical SEEG data recorded from 5 patients with drug-refractory epilepsy. Our method has been proven to not only achieve a higher level of accuracy and other aspects than existing studies, but also better balance sensitivity and specificity, making it more suitable for clinical application.

The main contributions of our study are summarized below:

1. Our study proposed a two-stage automatic detection method for HFOs. Specifically, in the first stage, an initial detector based on the threshold was designed to obtain the candidate event set of suspected HFOs, while in the second stage, based on the candidate set, we constructed a deep learning model for further detection.
2. To integrate the advantages of both modals' data, we proposed an end-to-end bi-branch fusion model, where two backbone networks (1d-ResNet + LSTM & 2d-ResNet_CBAM) are designed to learn deep features of filtered signals and time-frequency images, respectively. The results of ablation experiments demonstrate the effectiveness of the proposed method. And it has surpassed other reported methods in sensitivity, specificity, and other aspects.
3. We proposed 1d-ResNet + LSTM model in signal branch, where 1d-ResNet is responsible for extracting features in the signal morphological space, and LSTM focuses on the features in the time dimension of signals.
4. We proposed 2d-ResNet_CBAM model in TFpic branch, which can pay more attention to the useful information in images with adding spatial and channel attention mechanism to the baseline.

RETRACTED

The rest of this paper is organized as follows.  Section 2 demonstrates the materials and the proposed method.  Section 3 presents the experimental results and relevant comparison.  Section 4 analyzes and discusses the method and results, as well as the limitation and future works. Finally, Section 5 concludes this paper.

## 2. Materials and Methods

### 2.1. Materials

#### 2.1.1. Data Acquisition

The study involved 5 patients with drug-resistant epilepsy from Xuanwu Hospital of Capital Medical University. The detailed information is shown in Table 1. All patients have undergone preoperative routine scalp EEG examinations and various imaging examinations (including MRI and PET). At the same time, all patients were discussed by clinicians in a multidisciplinary manner. Combined with preoperative evaluation of the diagnosis results, electrode planning and stereotactic EEG were performed, which has been shown to be useful in identifying epileptic zones [37]. Specifically, enhanced thin-scan MRI (layer thickness 1 mm, interval 1 mm) and thin-scan CT (layer thickness 1 mm, interval 1 mm) were imported into a robotic stereotactic surgery assistant workstation (robotied stereotactic assistant, ROSA, from a French company named Medtech) for data fusion; then the electrode implantation plan was designed.

The SEEG electrode we used is 0.8 mm in diameter and each electrode has 5–18 contacts, each of which is 2 mm in length and 1.5 mm in spacing, as shown in Figure 1(a). A typical medial temporal lobe electrode reconstruction is shown as Figure 1(b). The long-range SEEG data of each patient is collected at a frequency of 2048 Hz, with files in .eeg format, and patients' video records can be viewed through Natus Neuroworks software. Based on the video records of each patient, we randomly select the SEEG records of each patient's waking interval and sleeping interval for 2 hours. The interval between the selected record and the patient's onset is at least 1 hour. The EDF format is exported, and the channel distribution of each patient is recorded at the same time. Noted that the data exported here has not been subjected to any preprocessing operations.

RETRACTED

#### 2.1.2. Data Preprocessing

The original interphase SEEG data of all subjects need to go through a preprocessing process, including data segmentation, polarity conversion, bad channels removal, band-pass filtering, notch filtering, etc. The overall process is shown in Figure 2. The collected SEEG were long-term records with large scale, in general; 2 hours of data occupies about 8 G of memory, but the computer and software can use limited memory. In theory, the segmenting signals could provide the same information as the longer records, so part of them needed to be intercepted for the experiment, and generally 30 min signal fragments were taken for subsequent operation. Normally, the waveforms and amplitudes of the bipolar data are less distorted, so it is necessary to perform polarity conversion operation on the original SEEG. Since some interference is often encountered in the process of EEG recording and some empty electrodes are often placed in clinical practice, we removed these obviously disturbed channels and empty electrodes before using. Moreover, signal acquisition equipment uses 50 Hz mains power supply; the 50 Hz frequency-doubling notch filter should be used to filter out the power-frequency interference and frequency-doubling interference. Finally, in view of the fact that the HFOs have greater energy in the frequency range of 80–500 Hz compared with the background signals, the signals ranging from 80 to 500 Hz are retained through the band-pass filter.

Several tools are involved in the preprocessing, such as AnyWave, EDFBrowser, and so on. Specifically, we use EDFBrowser to segment the discontinuous original EEG signals to obtain continuous signal fragments and then use AnyWave to perform polarity conversion, bad channels removal, band-pass filtering, and notch filtering.

#### 2.1.3. Artificial Visual Marking

In the two-stage automatic detection method, the data collected and preprocessed in the above process are screened by the initial detector to obtain the HFO candidate event set. Usually, there were a certain number of false positive samples in this candidate pool, namely, non-HFOS. In view of this, we further invited clinical experts to distinguish true or false HFOs and took the result as the gold standard of this study to construct our clinical private database.

The marking task is completed by two professional doctors. The frequency of the real HFOs in our database ranges from 80 to 500 Hz, of which the ripple frequency range is 80–250 Hz, and the fast ripple frequency range is 250–500 Hz. Besides, different kinds of artifacts are included in the HFO database, which are counted as non-HFOs. The marking process uses the original EEG data, the 80–500 Hz frequency band-pass signal, and the wavelet transform time-frequency diagram together as a reference. When the original signal has oscillations, and the signal amplitude after filtering is significantly higher than the baseline and there is an islanding effect in the time-frequency diagram meanwhile, it is considered that it meets the HFO signal standard, and it will be labeled and saved. On the contrary, the negative samples that do not meet the standard will be labeled and saved as well. Thus, the positive and negative sample data set is established.

RETRACTED

Figure 3 shows several typical signal waveforms. Among them, (a) and (b) are considered as real HFOs, while (c), (d), and (e) are 3 different types of artifacts, which constitute non-HFOs set. As we see, when filtering sharp transient signals (such as epileptic spikes, sharp waves, and sharp artifacts) or signals with harmonics, it may cause “false” high-frequency oscillation events, sharing similar waveforms in filtered signal with the real HFOs, as shown in the middle row, which makes the error of initial detector. However, these false events' time-frequency diagram is very different from that of real HFO events, as shown in the bottom row. Normally, spike-type artifacts usually caused by a band-pass filter tend to show a “candle-” like upward trend on the time-frequency diagram, while harmonic-type artifacts show dispersive high energy in the entire frequency range, while real HFO events often show the shape of “island” [38].

In order to ensure the objectivity and the efficiency, 2 doctors separately labeled a small number of samples as needed and then analyzed the labeling results of them and reached a unified labeling principle. Finally, all candidates were labeled. A total of 16167 records of positive and negative samples were generated, of which 7754 records were marked as positive samples and 8413 records were marked as negative samples.  Table 2 shows the details.

### 2.2. System Overview

The overall process of the proposed method of our study is shown in Figure 4. First, the patients' raw SEEG signals were collected and preprocessed including segmenting and filtering, etc., and the candidate event set of clinical high-frequency oscillation was preliminarily established by threshold detector. Then, the data was conducted by continuous wavelet transform (CWT) to generate 2d time-frequency images. Then, combined with three modes of data (the time-frequency diagram, the original signal, and the filtered signal), neurologist did the visual marking to distinguish true or false HFOs, and then we constructed our private data. Finally, we designed an end-to-end bi-branch fusion model for HFO automatic detection. Two modals' data were taken as the model input, and the hybrid network of 1d-ResNet and LSTM is constructed for signal branch, while 2d-ResNet with a CBAM followed is designed for TFpic branch. The feature learning of the two modals' data was carried out, and then we fused the output of the two parts by constructing a fusion module, in which the multilayer perceptron (MLP) classifier is used to recognize the results. A synchronous training strategy was adopted in the training process. After the training, the performance of the model was tested with test data and the classification results were evaluated.

RETRACTED

### 2.3. Initial Detector Based on Threshold Detection Method

In the first stage of our automatic detection method, an initial detector was designed, which can detect HFOs from a long-range recording as much as possible; that is, the algorithm should have the characteristics of high sensitivity and low specificity. In general, in the band-pass filtered signal, when there are at least 3 continuous peaks exceeding 3–5 standard deviations, the signal is considered to be a true HFO [39]. On the basis of the initial detection, the clinicians only need to do visual marking on the signal within the suspected event set. This method can improve the labeling efficiency of HFOs.

The initial detection algorithm based on threshold is as follows:

1. The standard deviation (SD) of each channel of the subject was calculated based on the filtered signals, 2.5 times of peak value was defined as the threshold, and the position where the peak value of each signal exceeded the threshold was counted.
2. The times of the crossover between threshold and peak value in each 128 sampling points were counted, and the positions where the crossover times are greater than 3 were recorded.
3. The signal envelope was extracted by the Hilbert transform, and the position exceeding the threshold was recorded by setting the 3 times of background median value as the threshold value.
4. For the position that simultaneously meets the above 3 requirements, signal fragments of 0.1 s before and 0.4 s after that point, a total of 0.5 s, are extracted as a suspected HFO.

Figure 5 shows an example of using this initial detection.

### 2.4. Bi-Branch Fusion Model

After the initial detector, we obtained an HFO candidate pool containing all the suspected HFO events. On the whole, both of the 80–500 Hz band-pass signal and 2d time-frequency diagram are taken as the model input. Then, two deep backbone networks (1d-ResNet + LSTM and 2d-ResNet_CBAM) were built for the two inputs, respectively, to extract the high-order features of different modal data. Specifically, the signal branch is designed as a hybrid network with a 1d-ResNet and a LSTM connected in parallel, while the TFpic branch is implemented using a 2d-ResNet with a CBAM module embedded behind each convolutional block. Then the two output vectors from each branch were fused. Finally, a multilayer perceptron was used as a classifier to classify true/false HFOs. The overall architecture of the bi-branch model is shown in Figure 6.

RETRACTED

#### 2.4.1. Signal Branch

In order to avoid low frequency interference [25] and the impact of a little amount of irrelevant frequency bands higher than 500 Hz on HFO detection [40, 41], we use band-pass filtered signals ranging from 80 to 500 Hz as the input data of the model.

The overall structure of the signal branch is shown in Figure 7. In the signal branch, we adopted a hybrid network based on a 1d-ResNet34 and LSTM, where they were connected in parallel to realize the deep feature learning from each branch.

(a) On one hand, the 1d-ResNet34 is used to model the morphological characteristics of the signal. We choose a kind of CNN (ResNet) with residual connection to achieve this purpose. In the residual network, it is assumed that the mapping relation to be solved is *H* (*x*) and then break it down into two parts, that is:
  (1) $$\begin{array}{c} H\left(x\right)=F\left(x\right)+x, \end{array}$$
where *F*(·) is the residual function [42]. Then, at the high level of the network, learning an identity mapping *H*(*x*)⟶*x* is equivalent to making the residual part approach 0, that is, *F*(*x*)⟶0. It can be implemented in the form of a tier-hop connection, in which the input of the element is directly added to the output of the element. Specifically, according to the 2d-ResNet proposed by He et al. [42], we rewrote it into a 1d version. The 1d-ResNet model consists of 5 stages. The first stage is a 7 × 7 convolution process, stride is 2, and then after pooling, the size of the feature map has become 1/4 of the input. Next are four stages of stacking of four residual blocks. ResNet34 uses the basic residual block defined by He et al. [42]. Each block is composed of two superimposed 3 × 3 convolutions. The number of block stacks is [3, 4, 6, 3].
(b) On the other hand, a kind of RNN (LSTM) that can learn temporal correlation is introduced into the network designing. Specifically, an LSTM block with 100 hidden units and 2 layers is used for feature extraction.
(c) On the basis of the spatial modeling of signals by CNN (1d-ResNet), supplemented by the temporal modeling by RNN (LSTM), a hybrid network is formed to model signal features from multiple perspectives. The higher order characteristic representation of the signal is obtained. Finally, the output vectors obtained from two dimension are fused and spliced to obtain the multiperspective fusion features of the filtered signals.

RETRACTED

#### 2.4.2. TFpic Branch

In order to enable the model to better learn the differences between the time-frequency image of real HFOs and non-HFOs, a TFpic branch is established.

First, we need to perform time-frequency transformation on the patient's filtered SEEG signal. Epilepsy EEG signals change both on the time scale and on the frequency scale and are a kind of random signal. The wavelet transform can perform multiresolution analysis of the signal, which is very suitable for feature extraction of random nonstationary EEG signals. Morlet wavelet is used here to transform the signal, and its wavelet basis function is as follows:

(2) $$\begin{array}{c} \Psi_{a,b}\left(t\right)=\exp\left(i\omega_{0}\frac{t-b}{a}\right)\exp\left(-\frac{{\left(t-b\right)}^{2}}{2a^{2}}\right), \end{array}$$

where *ω*_0_ represents the center frequency, *a* represents the stretching amount of the wavelet basis, and *b* represents the translation amount of the wavelet basis. Furthermore, according to the properties of Fourier transform, it can be deduced that the formula of wavelet transform is

(3) $$\begin{array}{c} \Psi f\left(a,b\right)=\int_{-\infty }^{+\infty }f\left(t\right){\bar{\psi }}_{a,b}\left(t\right)\text{d}t\\ =\int_{-\infty }^{+\infty }f\left(t\right)\exp\left(-i\omega_{0}\frac{\left(t-b\right)}{a}\right)\exp\left(-\frac{{\left(t-b\right)}^{2}}{2a^{2}}\right)\text{d}t. \end{array}$$

Secondly, we designed a deep backbone network for TFpic branch as shown in Figure 8. On the whole, this branch adopts 2d-ResNet as a baseline framework and adds a CBAM module to it. ResNet is a commonly used backbone network in image classification. As described before, it adds residual block into the classic CNN. On this basis, the study introduces the CBAM module to further improve the performance of the model.

Specifically, a 2d-ResNet50 is applied to feature extraction of the whole branch, and the whole model is composed of 5 stages. Different from signal branch, Resnet50 uses its own personalized residual blocks defined by He et al. [42]. Each block consists of 3 convolutional layers (1 ∗ 1, 3 ∗ 3, 1 ∗ 1) to compress dimensions, convolutional processing, and restore dimensions. The number of blocks stacked is [3, 4, 6, 3].

RETRACTED

Furthermore, CBAM is embedded after each block of the 2d-ResNet. In the channel attention (CA) module, the input feature graphs are, respectively, pored through global maximum pooling and global average pooling based on width and height and then, respectively, through MLP. The output features of MLP were added elementwise and then activated by sigmoid to generate the final CA feature map. It can be computed as proposed by Woo et al. [43]:

(4) $$\begin{array}{c} M_{c}\left(F\right)=\sigma \left(\text{MLP}\left(\text{AvgPool}\left(F\right)\right)+\text{MLP}\left(\text{MaxPool}\left(F\right)\right)\right)\\ =\sigma \left(W_{1}\left(W_{0}\left(F_{avg}^{c}\right)\right)+W_{1}\left(W_{0}\left(F_{\max}^{c}\right)\right)\right), \end{array}$$

where *σ* denotes the sigmoid function, *W*_0_ ∈ *ℝ*^*C*/*r*×*C*^ and *W*_1_ ∈ *ℝ*^*C*×*C*/*r*^ denote the MLP weights, which are shared for both inputs, and the ReLU activation function is followed by *W*_0_. In the spatial attention (SA) module, global maximum pooling and global average pooling of input are performed, respectively, based on channel, and then concat operation is performed along the channel dimension. Then via a convolution operation, the dimension is reduced to 1. Finally, through sigmoid, SA characteristic graph is generated. It can be computed as proposed by Woo et al. [43]:

(5) $$\begin{array}{c} M_{s}\left(F\right)=\sigma \left(f^{7\times 7}\left(\left[\text{AvgPool}\left(F\right);\text{MaxPool}\left(F\right)\right]\right)\right)\\ =\sigma \left(f^{7\times 7}\left(\left[F_{\text{avg}}^{s};\;F_{\max}^{s}\right]\right)\right). \end{array}$$

Finally, CA module and SA module are connected in series and embedded into the back of each block of 2d-ResNet50. The embedded network (2d-ResNet_CBAM) can effectively learn the information which is helpful to classification from the input image and suppress some unnecessary information meanwhile.

#### 2.4.3. Fusion Module

The core breakthrough of this study is to propose the fusion of filtered SEEG signals and time-frequency map features.

The overall structure of feature fusion module is shown in Figure 9. For a certain candidate event, the deep features of 80–500 Hz band-pass signal is obtained through the signal branch, and similarly, the time-frequency image is put into the TFpic branch to obtain image deep features. Then, we combine the features from 2 branches to get a fused output vector for this candidate event. Among them, the dimension of signal branch output is 1 ∗ 612, and the dimension of TFpic branch output is 1 ∗ 2048, so the fused output vector dimension is 1 ∗ 2660. After that, it was subsampled by 0.5 times to obtain 1 ∗ 1330-dimensional fused output vector of one candidate event.

RETRACTED

Finally, all HFO candidate events are fed into a multilayer perceptron for training, and the classification (real/non-HFO) of each event is obtained. The output of hidden (*H*) and output (*O*) layer can be computed as follows:

(6) $$\begin{array}{c} H=XW_{h}+b_{h},\\ O=HW_{o}+b_{o}\\ =XW_{h}W_{o}+b_{h}W_{o}+b_{o}, \end{array}$$

where *X* is input vector, *W*_*h*_ and *W*_*o*_ are the weight matrices of the hidden layer and output layer, and *b*_*h*_ and *b*_*o*_ are the bias of them.

Besides, during training, binary cross entropy loss function is used, and its definition is as follows:

(7) $$\begin{array}{c} L_{\text{logistic}}\left(\hat{y},y\right)=-y\;\log\hat{y}-\left(1-y\right)\log\left(1-\hat{y}\right), \end{array}$$

where *y* is the expected output, *y* ∈ {0,1}, and $\hat{y}$ is the actual output.

## 3. Results

### 3.1. Evaluation Metrics

In this work, we selected some indicators to evaluate the performance of the proposed model, mainly including accuracy (ACC), sensitivity (SEN), specificity (SPE), precision (PRE), false discovery rate (FDR), and F1-score. In addition, to illustrate that the proposed method achieves a better balance between sensitivity and specificity, we defined SEN_SPE-score.

Most indicators are calculated according to the confusion matrix. In the confusion matrix, true positive (TP) means that the predicted category and true category are consistent and both are *P*; on the contrary, true negative (TN) means that the predicted category and true category are both *N*. False positive (FP) means that the forecast category is *P*, but the true category is *N*, as opposed to false negative (FN) which means that the forecast category is *N*, but the true category is *P*. The specific calculation formula of these indicators is as follows:

(8) $$\begin{array}{c} \text{Accuracy}\left(\text{ACC}\right)=\frac{\text{TP}+\text{TN}}{\text{TP}+\text{FP}+\text{TN}+\text{FN}},\\ \text{Sensitivity}\left(\frac{\text{SEN}}{\text{recall}}\right)=\frac{\text{TP}}{\text{TP}+\text{FN}},\\ \text{Specificity}\left(\text{SPE}\right)=\frac{\text{TN}}{\text{TN}+\text{FP}},\\ \text{Precision}\left(\text{PRE}\right)=\frac{\text{TP}}{\text{TP}+\text{FP}},\\ F1\text{ score}=\frac{2^{*}{\text{Precision}}^{*}\text{Recall}}{\text{Precision}+\text{Recall}},\\ \text{FDR}=\frac{\text{FP}}{\text{TP}+\text{FP}}=1-\text{Precision}. \end{array}$$

Similarly, we calculate the harmonic mean of sensitivity and specificity (SEN_SPE-score) to measure the balance degree of the model on these two indicators, with the specific formula as follows:

(9) $$\begin{array}{c} \text{SEN}\_\text{SPE}-\text{score}=\frac{2*\text{SEN}*\text{SPE}}{\text{SEN}+\text{SPE}}. \end{array}$$

RETRACTED

### 3.2. Parameter Setting, Training Strategy, and Experiment Environment

The optimal values of all parameters used in the study are shown in Table 3.

In terms of the model design, in order to ensure the adequate model capacity and prevent overfitting meanwhile, we empirically set the LSTM hidden size as 100, the LSTM layers number as 2, and the number of hidden layer neurons in the fusion module as 500. In addition, the number of ResNet blocks stacked was set as [3, 4, 6, 3] in both of the signal branch and TFpic branch according to the classical design principles of ResNet.

In terms of the hyperparameters in network training, we selected the parameters of the initial learning rate, batch size, and training epochs as 0.01, 32, and 60, respectively. Specifically, the basis for hyperparameters selection is that when the model achieved the best result in the validation set, the values of each parameter were recorded. In our experiment, we divided the experimental data into training set, validation set, and test set, which will be shown in the next section. We trained the model on the training set, selected parameters according to the results of the validation set, and finally used the test set for testing to support our idea.

In our study, we used a bi-branch synchronous training strategy to feed the input of the band-pass filtered signal and time-frequency diagram into the model; that is, the input data of the bi-branch should be one-to-one correspondence. The input data of the two different modes are propagated backward and forward until the output generates errors, and then the errors are propagated back to update the weight matrix.

Our experimental environment is as follows. We conducted all of our experiments on the HP Z8G4 graphics workstation with a single Nvidia GeForce RTX 2080Ti and 12G graphic memory in the process of model training and testing.

### 3.3. Training and Testing Sets

In order to make full use of our database, each patients' record corresponds to 1 data subset, and the data set is divided into 5 folds to generate 5 groups of experimental data, and two validation methods are adopted, namely, intrasubject validation and cross-subject validation.

#### 3.3.1. Intrasubject Validation

The data partitioning and usage of the intrasubject validation are shown in Figure 10. Specifically, we selected 4 of 5 data subsets each time (a total of 5 groups of selection), then randomly shuffled, and then randomly selected 80% of the data as the training set, 10% of the data as validation set, and the remaining 10% of the data as the test set.

#### 3.3.2. Cross-Subject Validation

In this work, we made an important breakthrough in applying the model to cross-patient tests, which still achieved high performance. The specific results will be shown in the following sections.

RETRACTED

The specific data division and usage were shown in Figure 11. Specifically, we used the leave-one method for cross-validation, with each subset of the 5 subsets being used as the test set in turn and the remaining subset containing the other 4 patients in white background as the training set and validation set, where 80% of them is training set and 20% is the validation set. Five pretrain models were obtained with five different training sets, and performance tests were carried out on their respective test sets. Finally, the performance of the five groups of data were averaged.

### 3.4. Performance of Our Method

#### 3.4.1. Performance of Intrasubject Validation

We included the 5 clinical patients' SEEG record into the study and adopted the intrasubject validation to obtain the average sensitivity of 94.62%, average specificity of 92.70%, average precision of 92.12%, average accuracy of 93.62%, average FDR of 7.88%, average *F*1-score of 93.33%, and the average of SEN_SPE-score of 93.63%, as shown in Table 4.

#### 3.4.2. Performance of Cross-Subject Validation

In cross-subject validation, 5 groups of experiments were carried out. The results showed that the average sensitivity was 92.00%, the average specificity was 88.26%, the average precision was 86.86%, the average accuracy was 89.76%, the average FDR was 13.14%, the average F1-score was 89.11%, and the average of SEN_SPE-score was 89.87%, as shown in Table 5.

### 3.5. Comparison with Existing Methods

In this section, we compared the classification effectiveness of several reported HFO automatic detection methods. In order to display the comparative results objectively, we found that most of the studies randomly sampled all the labeled data without dividing them by patients, and some of the studies carried out cross-validation among patients. Therefore, the results of the two types of studies are shown in Tables 6 and 7.

Specifically, in terms of the intrasubject validation, the automatic HFO detector based on Gabor transform which was reported in 2016 achieved a sensitivity of 81.1% in ripples and 74.6% in fast ripples [44]. In more recent studies, the automatic detector using the combination of short-time energy and CNN reported in 2019 achieved a sensitivity of 91.26%, a specificity of 91.52%, and a precision of 88.67% in 2700 HFO events from 5 patients [21]. Sciaraffa et al. [27] proposed a new double-step machine learning method in 2020 to detect HFOs, which achieved a sensitivity of 87.40% and a specificity of 77.60%. Guo et al. [45] developed a hypergraph-based detector to automatically detect HFOs in 2021, which achieved an accuracy of 90.7%, a sensitivity of 80.9%, and a specificity of 96.9%. What is more, in 2021, Sharifshazileh et al. [46] presented a neuromorphic system that combines a neural recording headstage with a spiking neural network, which achieved a high sensitivity of 100% but a very low specificity of 33% and an accuracy of 78%.

RETRACTED

In terms of the cross-subject validation, in 2019, Zuo et al. [28] proposed to convert the collected candidate HFOs into a two-dimensional gray-scale matrix and then use a stacked CNN to further distinguish the candidate events, which achieved a sensitivity of 77.04% in ripples and 83.23% in fast ripples and a specificity of 72.27% in ripples and 79.36% in fast ripples. In 2021, Wu et al. [29] proposed a novel detector based on the stacked denoising autoencoder (SDAE) and the ensemble classifier with sample weight adjusting factors, which achieved a sensitivity of 92.4% in ripples and 90.3% in fast ripples and an FDR of 9.2% in ripples and 10.7% in fast ripples. Besides, in 2021, Wang et al. [47] proposed an algorithm to calculate the dynamic baseline based on the maximum distributed peak points to automatically detect HFOs and achieved a sensitivity of 82.666% and a specificity of 63.352%.

The proposed bi-branch feature fusion model combines the advantages of two types of input data; thus its sensitivity, specificity, and accuracy are better than the existing detectors, not only for the data divided randomly, but also for the data divided between patients. Our method has shown a good generalization performance and also has made a good balance of sensitivity and specificity compared to other existing methods with the highest SEN_SPE-score of 93.63% and 89.87%, respectively among them, which makes it of high clinical significance and research value.

### 3.6. Ablation Study

In this section, we focus on verifying the effectiveness of the bi-branch network, analyzing the role of each single branch. Specifically, two single-branch reference models are used to compare with the proposed model, TF-Branch means that only time-frequency diagrams of HFO candidates are used as network inputs, and Sig-Branch means that only band-pass filtered signals are fed into network. When training and testing the two single-branch models, the data set partition rules are consistent with the aforementioned cross-subject validation method; that is, the leave-one method is used for cross-validation.

For the TF-Branch model, the mean sensitivity was 69.01%, the mean specificity was 91.59%, the mean precision was 86.76%, the mean accuracy was 81.23%, the mean FDR was 13.24%, and the mean F1-score was 76.59%. For the Sig-Branch model, the mean sensitivity was 94.16%, the mean specificity was 80.65%, the mean precision was 80.52%, the mean accuracy was 86.81%, the mean FDR was 19.48%, and the mean F1-score was 86.69%. The details are shown in Table 8.

RETRACTED

Figure 12 shows the classification performance of the three models. Note that the sensitivity and specificity of the two single-branch models were higher than those of the bi-branch model, respectively. The specificity of the TF-Branch model was 3.33% higher than that of the proposed method, and the sensitivity of the Sig-Branch model was 2.17% higher than that of the bi-branch model.

However, in clinical application, sensitivity and specificity are equally important. Neither miss diagnosis nor misdiagnosis can be tolerated. Ideally, we should find a balance between them.

For the TF-Branch model, the SEN_SPE-score is 78.71%, while the Sig-Branch model is 86.88%. Specially, the SEN_SPE-score of the bi-branch model proposed in this paper is 90.09%, which is 7.29% higher than that of the other two single-branch models. It can be seen that although the proposed model has a tiny loss on a single indicator, it greatly balances the SEN and SPE, making it more suitable for aiding clinical diagnosis.

What is more, in addition to the SEN and SPE, the other four indicators have been improved significantly by the proposed model. Among them, the precision increased by 3.22%, the accuracy increased by 5.73%, the FDR decreased by 3.22%, and the F1-score increased by 7.47%, which is shown in Table 9 in particular.

## 4. Discussion

### 4.1. Main Contribution of Our Study

Visual assessment is still the gold standard for clinical analysis of HFOs. Experts can visually mark the high-frequency oscillating rhythm in the EEG of patients according to their experience. However, due to the complicated process of visual labeling and the strong subjectivity and inconsistency among experts, it is necessary to develop a new automatic detection method. Since 2002, different HFO automatic detection methods have been reported in different studies. Our work has made further improvement and innovation on the basis of predecessors. Its main contribution lies in the following three aspects.

#### 4.1.1. Bi-Branch Fusion Model Realizes Complementary Advantages

The detectors proposed in the early usually use the EEG signal waveform, extract features, and then realize automatic classification. However, there are many artifacts and other signals in the band-pass filtered signals that cannot be distinguished from the real HFOS, so this leaves the problem of poor specificity and is prone to misdiagnosis in clinical practice. This problem can be solved by time-frequency diagrams, but the classification of signals only from the perspective of images usually gets a poor sensitivity and it is easy for it to miss diagnosis in clinical practice, so it is not suitable for practical clinical application.

RETRACTED

In order to solve this pain point, we innovatively proposed to use the filtered band-pass signal and time-frequency image as the input data of the model, establish a bi-branch deep learning model, fuse the output of the two branches, and then automatically classify HFOs/non-HFOs.

In the signal branch, the hybrid network (1d-ResNet + LSTM) combines the advantages of CNN and RNN. CNN is responsible for extracting features in the signal morphological space, and RNN is responsible for extracting features in the time dimension of signals, or it can be said that RNN is responsible for “memory.” In the TFpic branch, the 2d-ResNet_CBAM model paid more attention to the useful information of the time-frequency image, which can learn differences between the time-frequency diagram of real HFOs and non-HFOs.

By conducting the ablation experiment, we found that signal branch can achieve a high sensitivity but low specificity; on the contrary, TFpic branch can achieve a high specificity but low sensitivity. That is because, in filtered signals, the model is prone to errors in the resolution process due to the similar waveforms between positive and negative samples, while in time-frequency images, the obvious differences between positive and negative samples can make up for the low specificity of signal branches. However, in the time-frequency images, some true HFOs' time-frequency images may not have obvious islanding effect, but the filtered signal has obvious peak value higher than the background. As a result, when we combine these two branches, we can get a model with complementary advantages. It is illustrated that our study verified that information of filtering signals and time-frequency graphs should be taken into account in the analysis of HFOs.

Intuitively, results show that our strategy can effectively achieve the balance between sensitivity and specificity; at the same time, compared with other detectors, our method had higher accuracy and lower FDR. In addition, our study provides an end-to-end detection method; each branch automatically learns the higher order characteristics of two modal data, without feature extraction manually.

#### 4.1.2. Good Cross-Validation Supports Generalization Performance

In early studies, researchers mostly focused on the performance of signal detection, so in terms of dividing experimental data, most of them randomly divide training set and test set from the candidate pool [21, 27, 43, 45, 46]. In clinical application, when considering a new patient, it is desirable to transfer the a priori knowledge learned from previous existing cases to the judgment of the new patient. Therefore, the model must take into account the generalization ability between different patients. In the intrasubject validation mentioned above, data leakage is inevitable; that is, the same patient's data appears in both the training set and the test set. This method can check the model's performance to some extent, but since the data is not completely “unseen,” when the model is applied to a new patient, it is likely that there will be a significant performance deterioration that will not be able to meet clinical needs.

RETRACTED

In our research, we took the actual situation into consideration, so we adopted the leave-one method to cross-validate by dividing all data according to patients, so that the training set and the testing set are absolutely “unseen.” The results show that our detector is still well-performed even if in cross-validation, and all indicators are better than those of the same type of studies [28]. With the strong generalization performance, it makes our method more suitable as an auxiliary tool for clinical diagnosis.

#### 4.1.3. Automation Is Helping Healthcare

Our research is of great significance in practical clinical applications. In the aspect of individual diagnosis and treatment, when manual diagnosis is still the gold standard, misdiagnosis and missed diagnosis inevitably occur. Artificial intelligence technology hopes to help doctors by means of automation and provide more objective information to assist doctors in making judgments, so as to reduce errors to a certain extent. At the national development level, new technologies of automation can provide effective guidance and help for clinical undertakings in developing countries and promote social development.

### 4.2. Consistency Check between Visual and Automated Detection Results

In clinical application, HFO visual marking by doctors is used as the gold standard of this study. Therefore, we hope that the proposed detection method is highly consistent with the gold standard, so as to illustrate the effectiveness of the proposed method.

Cohen's kappa coefficient can be used to measure the consistency between different methods. It is calculated according to the confusion matrix, and the specific calculation formula is as follows:

(10) $$\begin{array}{c} \text{kappa}=\frac{p_{0}-p_{e}}{1-p_{e}}, \end{array}$$

where *p*_0_ is total accuracy, *p*_*e*_=(*a*_0_*∗b*_0_+*a*_1_*∗b*_1_)/*n∗n*, *a*_0_ and *a*_1_ are the quantities predicted by the model to be 0/1, and *b*_0_ and *b*_1_ are the actual quantities of the two classes 0/1. Its value ranges from −1 to 1, but usually between 0 and 1. It can be divided into five groups to indicate different degrees of consistency: 0.0∼0.20 indicates very low consistency, 0.21∼0.40 is fair, 0.41∼0.60 is moderate, 0.61∼0.80 stands for high consistency, and 0.81∼1 is for almost perfect.

RETRACTED

In this study, we calculated Cohen's kappa coefficient between the new detection method and the gold standard. The coefficients of the first group to the fifth group were 0.784, 0.765, 0.708, 0.957, and 0.762, respectively, with an average kappa coefficient of 0.795. It can be seen that the test results of the method proposed in this paper are highly consistent with doctors' judgment.

Kappa coefficient reflects the effectiveness of the proposed method from the overall perspective.  Figure 13 shows the comparison between the automatic test results of patient 4 and the clinician's judgment more intuitively. The horizontal axis shows the number of patient channels included in the study, and the vertical axis shows the number of HFOs/non-HFOs. It can be seen that our proposed method shows good consistency compared to the gold standard in each channel of the patient.

### 4.3. Limitations of Our Study and Future Work

In general, we used a small amount of data to validate the proposed model. However, there are several limitations in our work.

First of all, the patterns of abnormal discharge vary among epilepsy patients with different diseases. The data of 5 patients used in this study were from patients with hippocampal sclerosis (HS) epilepsy, whose discharge mechanism and manifestations were different from those of other types of epilepsy. For example, patients with focal cortical dysplasia (FCD) exhibit high-frequency oscillations as polyspikes [48] or rhythmic epileptiform discharges [49]. Therefore, we are not sure whether our model can be well applied to other types of patients, given the limitations of the disease type. In the following studies, we will collect more data of epilepsy patients with other pathological phenotypes and carry out more experiments.

Secondly, the network structure and modules we used are classic structure. Better feature extraction baselines and some enhanced variants of LSTM networks have been proposed to be more effective in other applications. So, some newer attempts using new networks and attention units are under way.

Thirdly, we find that there is still a certain degree of discrepancy between the automatic detection result and the diagnosis result of the clinician, which indicates that the technical solution needs to be further developed. Since clinicians cannot be replaced by artificial intelligence, it is very necessary to put professional authority in the hands of clinicians when the diagnosis of machine is different from that of clinicians. In the future work, we will use the clinician's diagnostic experience as an optimization of deep learning methods to continuously improve the technical solutions.

RETRACTED

Finally, the spatial differences of HFOs distribution can reflect the transmission of electrophysiological signals in epilepsy to some extent, and exploring this content is the premise of further exploring the pathological mechanism of epilepsy. However, analysis of spatial differences of epileptic regions using EEG signals alone is challenging and inaccurate and often requires a combination of other analytical methods, such as brain networks. We are currently conducting in-depth research and a large number of experiments on the distribution and propagation of HFO on different channels. It will be further reported in future studies.

## 5. Conclusions

Our study shows that the bi-branch model based on the two modal data can be used as a high sensitivity and high specificity automatic detection tool for HFOs, with good generalization performance among different patients. Therefore, the proposed method is very suitable for clinical application. Following advantages are mainly realized: (1) In terms of the model design, the proposed bi-branch model combines the advantages of SEEG signal and time-frequency image for HFOs detection and uses two independent backbone networks (1d-ResNet + LSTM and 2d-ResNet_CBAM) to extract the features of the two modes automatically and simultaneously. By making a fusion of two branches' output, the method achieves high classification accuracy, sensitivity, and specificity; (2) in terms of clinical application, the clinical validation of both the intrasubject validation and the cross-subject validation was carried out in our study. Specially, for the research using the cross-subject validation, our proposed method reached a good performance with high accuracy, sensitivity, specificity, etc. which makes it sufficient for practical clinical applications.

## Figures and Tables

**Figure 1:** SEEG deep brain electrode. (a) SEEG electrode. (b) Schematic diagram of typical medial temporal lobe electrode reconstruction.

**Figure 2:** Data preprocessing. (a) Process of data preprocessing. (b) Results of data preprocessing, the upper row shows the waveform before preprocessing, and the waveform after preprocessing lies below. Details in the red box are shown on the right column.

RETRACTED

**Figure 3:** Visual marking example. The upper row is the raw data, filtered signal (80–500 Hz) lies in the middle row, and the time-frequency diagram is shown at the bottom row. (a) Ripple; (b) fast ripple; (c) artifact 1, high frequency transients caused by a band-pass filter; (d) artifact 2, the amplitude is larger than the global background but not significantly different from the local activity; (e) artifact 3, harmonics of low frequency nonsinusoidal signals.

**Figure 4:** Process diagram of the proposed method: (a) data acquisition and preprocessing. (b) Initial detection and CWT. (c) Deep backbones for feature extraction. (d) Fusion module and classification.

**Figure 5:** An example of initial detection: (a) raw data. (b) Filtered band-pass signal (80–500 Hz). (c) Hilbert transform envelope graph, in which the median value of background activity is marked by the red line, and the black box shows the exceeding part. (d) The black box shows the initial detection result.

**Figure 6:** Overview of the bi-branch feature fusion model. (a) Multimodal input. (b) Deep backbone networks. (c) Feature fusion module and classification.

**Figure 7:** Structure of signal branch model. (a) Filtered band-pass signal. (b) The specific structure of 1d-ResNet + LSTM.

**Figure 8:** Structure of TFpic branch model. (a) Time-frequency diagrams. (b) The specific structure of 2d-ResNet_CBAM. (c) CBAM, the upper row shows the channel attention (CA) module, and the spatial attention (SA) module lies in the bottom row, *S* denotes the sigmoid function.

**Figure 9:** Structure of the feature fusion module.

**Figure 10:** Intrasubject validation.

**Figure 11:** Cross-subject validation.

**Figure 12:** Classification performance of three structures on average. (a) SEN, SPE, PRE, ACC, F1; (b) FDR.

**Figure 13:** Comparison between the automatic test results and the clinician's judgment on patient 4. (a) Automatic detecting result. (b) Visual marking result.

**Table 1:** Clinical characteristics of 5 patients.

Patient no., gender	Age	Epilepsy duration	Surgical pathology	Implantation sites	No. of selected/total channels (*n*)
Pt1, male	21	7	HS	LH, LA, LBF, LIF	14/78
Pt2, female	33	5	HS	LH, LA, LBF, LIF, RH	24/77
Pt3, female	36	20	HS	LH, LA, LFO, LAT, RH	17/84
Pt4, male	33	7	HS	RH, RA, RBF	19/77
Pt5, female	38	23	HS	LH, LA, LOF, LFO, RH	15/84
Mean ± SD	32 ± 6	12 ± 8	—	—	18 ± 4/80 ± 3

Surgical pathology: HS, hippocampal sclerosis. Implantation sites: LH, left hippocampus; LA, left amygdala; LBF, left basis frontal; LIF, left inferior frontal; LFO, left frontoparietal operculum; LAT, left anterior temporal; LOF, left orbitofrontal; RH, right hippocampus; RA, right amygdala; RBF, right basis frontal. No. of selected/total channels (*n*): number of epileptogenic channels/total number of recorded channels.

RETRACTED

**Table 2:** Clinical database of HFOs.

Patient no.	Data batch^1^	Positive^2^	Negative^3^	Total
Pt1	1	2905	2916	5821
Pt2	1	2411	2343	4754
Pt3	1	401	517	918
	2	412	604	1016
Pt4	1	412	555	967
	2	488	508	996
Pt5	1	225	533	758
	2	500	437	937
Total	—	7754	8413	16167

^1^Data batch represents different batches/times of data collection. ^2^Number of positive samples. ^3^Number of negative samples.

**Table 3:** Training parameters.

Step	Parameters	Setting
Signal branch	LSTM hidden size	100
	LSTM num layers	2
	Numbers of blocks stacked	[3, 4, 6, 3]

TFpic branch	Numbers of blocks stacked	[3, 4, 6, 3]

Fusion module	MLP number of hidden layer neurons	500

Overall	Initial learning rate	0.01
	Batch size	32
	Training epochs	60

**Table 4:** The results for the bi-branch feature fusion model using intrasubject validation.

Group	Confusion matrix						Evaluation metrics (%)		
	TN	FP	FN	TP	SEN	SPE	PRE	ACC	FDR	F1	SEN_SPE
1	698	57	34	657	95.08	92.45	92.02	93.71	7.98	93.52	93.75
2	692	49	47	631	93.07	93.39	92.79	93.23	7.21	92.93	93.23
3	675	69	21	657	96.90	90.73	90.50	93.67	9.50	93.59	93.71
4	1232	130	74	1126	93.83	90.46	89.65	92.04	10.35	91.69	92.11
5	546	20	27	440	94.22	96.47	95.65	95.45	4.35	94.93	95.33
Average					94.62	92.70	92.12	93.62	7.88	93.33	93.63

**Table 5:** The results for the bi-branch feature fusion model using cross-subject validation.

Group	Confusion matrix						Evaluation metrics (%)		
	TN	FP	FN	TP	SEN	SPE	PRE	ACC	FDR	F1	SEN_SPE
1	838	132	50	675	93.10	86.39	83.64	89.26	16.36	88.12	89.62
2	954	109	120	780	86.67	89.75	87.74	88.33	12.26	87.20	88.18
3	865	256	30	783	96.31	77.16	75.36	85.21	24.64	84.56	85.68
4	2282	61	41	2370	98.30	97.40	97.49	97.85	2.51	97.89	97.85
5	2642	274	418	2487	85.61	90.60	90.08	88.11	9.92	87.79	88.04
Average					92.00	88.26	86.86	89.76	13.14	89.11	89.87

**Table 6:** The comparison between proposed method and existing methods using intrasubject validation.

Methods	SEN (%)	SPE (%)	PRE (%)	ACC (%)	FDR (%)	F1 (%)	SEN_SPE (%)
[44]	81.1 (R)	—	—	—	30.2 (R)	—	—
	74.6 (FR)				6.3 (FR)		
[21]	91.26	91.52	88.67	—	—	89.95	91.39
[27]	87.40	77.60	—	—	—	—	82.21
[45]	80.9	96.9	—	90.7	—	—	88.18
[46]	100	33	—	78	—	—	49.62
Proposed	94.62	92.70	92.12	93.62	7.88	93.33	93.63

**Table 7:** The comparison between proposed method and existing method using cross-subject validation.

Methods	SEN (%)	SPE (%)	PRE (%)	ACC (%)	FDR (%)	F1 (%)	SEN_SPE (%)
[28]	77.04 (R)	72.27 (R)	—	—	—	—	74.58 (R)
	83.23 (FR)	79.36 (FR)					81.25 (FR)
[29]	92.4 (R)	—	—	—	9.2 (R)	—	—
	90.3 (FR)				10.7 (FR)		
[47]	82.666	63.352	—	—	—	—	71.73
Proposed	92.00	88.26	86.86	89.76	13.14	89.11	89.87

RETRACTED

**Table 8:** Classification performance with different structures.

Group	Model	Confusion matrix					Evaluation metrics (%)				
		TN	FP	FN	TP	SEN	SPE	PRE	ACC	FDR	F1
1	Bi-	838	132	50	675	93.10	86.39	83.64	89.26	16.36	88.12
	TF-	866	104	254	471	64.97	89.28	81.91	78.88	18.09	72.46
	Sig-	768	202	69	656	90.48	79.18	76.46	84.01	23.54	82.88

2	Bi-	954	109	120	780	86.67	89.75	87.74	88.33	12.26	87.20
	TF-	980	83	429	471	52.33	92.19	85.02	73.92	14.98	64.79
	Sig-	886	177	92	808	89.78	83.35	82.03	86.30	17.97	85.73

3	Bi-	865	256	30	783	96.31	77.16	75.36	85.21	24.64	84.56
	TF-	974	147	243	570	70.11	86.89	79.50	79.83	20.50	74.51
	Sig-	815	306	22	791	97.29	72.70	72.11	83.04	27.89	82.83

4	Bi-	2282	61	41	2370	98.30	97.40	97.49	97.85	2.51	97.89
	TF-	2308	35	363	2048	84.94	98.51	98.32	91.63	1.68	91.14
	Sig-	2098	245	18	2393	99.25	89.54	90.71	94.47	9.29	94.79

5	Bi-	2642	274	418	2487	85.61	90.60	90.08	88.11	9.92	87.79
	TF-	2656	260	793	2112	72.70	91.08	89.04	81.91	10.96	80.05
	Sig-	2288	628	174	2731	94.01	78.46	81.30	86.22	18.70	87.20

**Table 9:** The range of gains and losses in various indicators.

Methods	SEN	SPE	PRE	ACC	FDR	F1
Loss^1^	2.17%	3.33%	—	—	—	—
Improvement^2^	—	—	3.22%	5.73%	3.22%	7.47%

^1^Loss degree of SEN and SPE using bi-branch model compared with 2 single-branch models. ^2^Improvement degree of SEN and SPE using 2 single-branch models compared with the bi-branch model.

## Data Availability

The data used to support the findings of this study are available from the authors upon request.
